The article "Identification of the Vas Deferens in Laparoscopic Inguinal Hernia Repair Surgery Using the Convolutional Neural Network" was published in 2021. Journal: J Healthc Eng.

# Identification of the Vas Deferens in Laparoscopic Inguinal Hernia Repair Surgery Using the Convolutional Neural Network

**DOI:** 10.1155/2021/5578089

**Published:** 2021-09-22

**Authors:** Peng Cui, Song Zhao, Wenxi Chen

**Affiliations:** ^1^Biomedical Information Engineering Lab, The University of Aizu, Aizuwakamatsu, Japan; ^2^Department of General Surgery, People's Hospital of Hannan District, Hannan District, Wuhan, China

## Abstract

Inguinal hernia repair is one of the most frequently conducted surgical procedures worldwide. Laparoscopic inguinal hernia repair is considered to be technically challenging. Artificial intelligence technology has made significant progress in medical imaging, but its application in laparoscopic surgery has not been widely carried out. Our aim is to detect vas deferens images in laparoscopic inguinal hernial repair using the convolutional neural network (CNN) and help surgeons to identify the vas deferens in time. We collected surgery videos from 35 patients with inguinal hernia who underwent laparoscopic hernia repair. We classified and labeled the images of the vas deferens and used the CNN to learn the image features. Totally, 2,600 images (26 patients) were labeled for training and validating the neural network and 1,200 images (6 patients) and 6 short video clips (3 patients) for testing. We adjusted the model parameters and tested the performance of the model under different confidence levels and IoU and used the chi-square to analyze the statistical difference in the video test dataset. We evaluated the model performance by calculating the true positive rate (TPR), true negative rate (TNR), accuracy (ACC), positive predictive value (PPV), and *F*1-score at different confidence levels of 0.1 to 0.9. In confidence level 0.4, the results were TPR 90.61%, TNR 98.67%, PPV 98.57%, ACC 94.61%, and *F*1 94.42%, respectively. The average precision (AP) was 92.38% at IoU 0.3. In the video test dataset, the average values of TPR and TNR were 90.11% and 95.76%, respectively, and there was no significant difference among the patients. The results suggest that the CNN can quickly and accurately identify and label vas deferens images in laparoscopic inguinal hernia repair.

## 1. Introduction

Inguinal hernias are found in 3%–8% of the general population [1]. Inguinal hernia repair (IHR) is one of the most commonly used surgical methods in general surgery. More than 20 million inguinal or femoral hernias are repaired every year, and 75% of abdominal wall hernias are classified as inguinal hernia [2, 3].

With the development of medical technology and medical equipment, minimally invasive surgery has been performed widely. Transabdominal preperitoneal (TAPP) [4] and total extraperitoneal (TEP) [5] surgeries are the most commonly used minimally invasive methods for inguinal hernia.

The article "Identification of the Vas Deferens in Laparoscopic Inguinal Hernia Repair Surgery Using the Convolutional Neural Network" was published in 2021. Journal: J Healthc Eng.

However, laparoscopic IHR is considered to be technically challenging. Laparoscopic minimally invasive surgery method can reduce the extent of skin incisions, nerve damage, and hematoma; lower postoperative pain and risk of infection of the surgical site; and lead to quicker recovery [6, 7], but it also has several disadvantages: for example, the surgeon initially needs a longer surgery time before plateauing on his/her learning curve; the surgery has a higher risk of complications; it needs much more knowledge of pelvic anatomy; and it needs a high level of surgical skill [8, 9], which can lead to more mistakes and harm to patients during the learning process. In clinical practice, young surgeons need a long learning curve to carry out laparoscopic repair surgery well, especially TEP technology. With the increase of surgical experience and familiarity with local anatomy, complications and recurrence rates will gradually decrease [10].

Common complications of the operation include bleeding; bladder lesions; intestinal obstructions; intestinal perforations; injury to the iliac vein, femoral nerve, and vas deferens; and even death [8].

With the development of artificial intelligence (AI) technology, CNNs have become an effective method for medical image analysis, disease prediction and diagnosis, and lesion detection and have been widely used [11–13]. CNNs are not a solution to replace doctors, but will help doctors optimize their routine tasks, thus having a potentially positive impact on medical practice [14]. We have also applied deep learning technology to nerve and dura mater recognition under spinal endoscopy and achieved satisfactory results [15].

There are many neural network models for object detection [16–19], but each neural network has its own advantages. Some can detect objects quickly, but the precision is not optimal, while others can detect an object with higher precision, but the speed of detection is quite slow. In this research, we want to use a CNN model that can detect objects fast enough to be used at 30 frames per second and have good precision. YOLO is a one-stage convolutional neural network for object detection [20, 21], whose rate of detection can reach 65 fps with an average precision of up to 43.5% on the COCO dataset [21]. The innovations of this article are as follows: (1) combined with computer CNN technology and clinical data, a new method for identifying vas deferens images in laparoscopic inguinal hernia repair using the CNN model is proposed, and the object detection ability of the CNN model (YOLOv4) on the medical dataset is also tested; (2) different annotation methods are used to train the CNN model and to examine the performance of the model in the process of training and testing; (3) discussed with clinical experts and selected the appropriate IoU value to evaluate the performance of the model for reference by clinical surgeons.

The article "Identification of the Vas Deferens in Laparoscopic Inguinal Hernia Repair Surgery Using the Convolutional Neural Network" was published in 2021. Journal: J Healthc Eng.

## 2. Materials and Methods

### 2.1. Data Collection

This research was approved by the Ethics Committee at Hannan Hospital, Hannan District, Wuhan City, Hubei Province, China.

In this study, 35 adult male patients with inguinal hernia disease admitted to the hospital for laparoscopic surgery from April 2018 to December 2019 were selected. The laparoscopic image device used was KARL STORZ Endoscopy (22202020-110), America. All patients underwent laparoscopic hernia repair and signed a patient consent form. We collected information such as gender, age, disease name, and interoperation videos. All endoscopic surgeries were performed by senior endoscopic experts at Hannan Hospital. Details of the dataset are shown in Table 1, and the patient age distribution is shown in Figure 1.

#### 2.1.1. Inclusion Criteria

We selected those subjects satisfying all of the following three criteria: (i) adult male; (ii) the patient was diagnosed with inguinal hernia and underwent hernia repair for the first time; and (iii) the patient agreed to allow the use of video recordings for scientific research.

#### 2.1.2. Exclusion Criteria

We excluded subjects matching any of the following three criteria: (i) female patient; (ii) patients with irreducible inguinal hernia; and (iii) the laparoscopic surgery was converted into an open surgery for any reason.

### 2.2. Data Processing

The patients were randomly divided into three groups, 26 patients in the training dataset, 6 patients in the image test dataset, and 3 patients in the video test dataset. In the training dataset and image test dataset, we used MATLAB (9.6.0.1174912 (R2019a) Update 5, academic use) to decompose the surgical videos into images according to different datasets and then saved them. A laparoscopic expert selected these images manually; then, the other laparoscopic expert verified them and finally deleted the disputed images and reached an agreement. In the video test dataset, we selected two short video clips from each patient's full surgical video, each of which is 30 seconds. All the videos used in this study were 30 frames per second. One of them is a clip with the vas deferens image, and the other is a clip without the vas deferens image. Then, two laparoscopic experts verified these video clips and reached an agreement.

The article "Identification of the Vas Deferens in Laparoscopic Inguinal Hernia Repair Surgery Using the Convolutional Neural Network" was published in 2021. Journal: J Healthc Eng.

In order to balance the training data, we selected 100 images containing the vas deferens for each patient in the training dataset. In the image test dataset, we chose 200 images for each patient (100 images that included the vas deferens and 100 images without the vas deferens). Thus, a total of 3800 pictures (2600 images in the training dataset and 1200 images in the image test dataset) of the vas deferens and 180 seconds (90 seconds with the vas deferens and 90 seconds without the vas deferens) of video clips were chosen to form an experimental database. There was no overlap in patients and images between the training dataset, image test dataset, and video test dataset.

All the training data were labeled using software LabelImg (v1.8.1) and then validated by two laparoscopic experts; none of the researchers had any objection to the labeling results. The research flowchart is shown in Figure 2. The original images with the vas deferens, labeled images, and original images without the vas deferens are depicted in Figure 3.

### 2.3. Training Parameters and Computer Configuration

In order to achieve higher accuracy with a faster processing speed, we used a one-stage neural network, YOLOv4 (based on the Darknet framework), to train and test the above datasets.

For training the model, we randomly divided the training dataset (2,600 images) into training data and internal validation data according to the ratio of 9 : 1. The details of neural network training parameters are as follows: input size = 416 ∗ 416, batch = 64, subdivisions = 32, initial learning rate = 0.001, momentum = 0.95, and max-batches = 10000.

Because our study is only a binary classification task, vas deferens tissue will only appear in one area of an image in laparoscopic IHR. Therefore, in the target detection stage, we adjusted the parameters in the process of nonmaximum suppression (NMS) and set NMS-IoU to 0.1 to reduce the number of detection boxes.

The computer was an Intel i9 9900k CPU @3.6 GHz × 16, RAM 32 GB, with a CUDA-enabled Nvidia Titan 312 GB graphics processing unit (Nvidia), based on hardware of the NVIDIA GeForce RTX 2070 SUPER GPU. The whole training time was about 12 hours.

## 3. Results

We examined the test dataset using the best training weight in the training process, and then two laparoscopic experts verified whether the images in the test dataset were correctly labeled by the model. The two laparoscopic experts verified the labels in all the images and further discussed any labeled images that were controversial. Finally, they reached an agreement on all the labeling results.

We defined those images with the vas deferens that were correctly labeled as true positive (TP); the images without the vas deferens but wrongly identified and labeled incorrectly as false positive (FP); the images containing the vas deferens but not identified and not labeled as false negative (FN); and the images without the vas deferens and without any label as true negative (TN).

The article "Identification of the Vas Deferens in Laparoscopic Inguinal Hernia Repair Surgery Using the Convolutional Neural Network" was published in 2021. Journal: J Healthc Eng.

In the image test dataset, we used different confidence levels from 0.1 to 0.9 to evaluate the performance of the model. The model was used to label the images in the image test dataset, and two laparoscopic experts examined these results. For 600 positive symbols (images include the vas deferens), a total of 607 detection boxes were labeled on these images. The detailed test results at different confidence levels are shown in Table 2. Example images of TP, FP, and FN are shown in Figure 4.


(1) $$\begin{array}{c} \mathrm{TPR}=\frac{\mathrm{TP}}{\left(\text{TP}+\text{FN}\right)}\text{ ,}\\ \mathrm{TNR}=\frac{\mathrm{TN}}{\left(\mathrm{TN+FP}\right)},\\ \mathrm{PPV}=\frac{\mathrm{TP}}{\left(\mathrm{TP+FP}\right)},\\ \mathrm{ACC}=\mathrm{TP+}\frac{\mathrm{TN}}{\left(\mathrm{TP+TN+FP+FN}\right)},\\ F1=\frac{2*\text{PPV}*\text{TPR}}{\left(\text{PPV}+\text{TPR}\right)}. \end{array}$$

According to the test results in Table 2, we used the following indicators to evaluate the performance of the CNN model: true positive rate (TPR), true negative rate (TNR), accuracy (ACC), positive predictive value (PPV), intersection over union (IoU), average precision (AP), and *F*1-score. We also draw the receiver operating characteristic (ROC) curve and calculate the AUC value as indicators to evaluate the performance of the model. The formulas used to calculate these values are as follows, and the results are shown in Table 3. The ROC curve is shown in Figure 5. The performance of the model for different IoUs is shown in Table 4.

According to the ROC curve, we calculate that the optimal confidence threshold of the model is around confidence level 0.4, and the AUC value is 0.97, so in the process of testing the video test dataset, we use the confidence level of 0.4 to test the real-time detection function of the model. After saving the video detection results, we decompose the video clips into images for verification. A total of 5433 images were decomposed from the video clips (2719 with the vas deferens and 2714 without the vas deferens). Two laparoscopic experts verified these images one by one and confirmed the results. The evaluation indicators and specific results are shown in Table 5.

In the video test dataset, these results were analyzed using IBM SPSS Statistics version 23.0. We used the chi-square test to analyze the statistical differences between patients, with *p* > 0.05, meaning no significant difference between the tested objects. The *p* value of TPR was 0.768, the *p* value of TNR was 0.608, and all *p* values were greater than 0.05; the average TPR, TNR, PPV, and ACC were 90.11%, 95.76%, 95.52%, and 92.93%, respectively. The results show that the model can effectively identify the vas deferens images in laparoscopic inguinal hernia repair, and the sensitivity and specificity of the model to different patients in the video test dataset are not statistically different.

The article "Identification of the Vas Deferens in Laparoscopic Inguinal Hernia Repair Surgery Using the Convolutional Neural Network" was published in 2021. Journal: J Healthc Eng.

We also tested the real-time detection ability of the model. The results show that when the input size is 416 ∗ 416, the detection speed of the model can reach 45.32 frames per second, and the detection speed is greater than 30 frames per second, which meets the real-time detection requirements of laparoscopic inguinal hernia repair.

## 4. Discussion

Using CNNs for medical image detection is not new, but using this technology to detect the vas deferens under laparoscopic IHR surgery is novel; we use the CNN model to train and test the vas deferens images and obtained good results.

### 4.1. Performance of the CNN-Based Identification

In order to select the appropriate parameters and indicators to evaluate the performance of the model, we set different confidence levels to calculate the evaluation indicator. Laparoscopic experts verified the labeled images one by one and concurred on the final results.

According to Table 3, it is clear that, with increasing confidence levels, TPR gradually decreased from 95.06% to 75.95%, while TNR and PPV gradually increased from 90.67% and 91.15%, respectively, to 100%. In order to observe the performance of the model more comprehensively, we also calculated the ACC and *F*1-score, both of which first increased and then decreased with increasing confidence levels.

The *F*1-score is often used as a comprehensive index to judge the performance of a CNN model; it is a combination of TPR and PPV. When the confidence level is 0.2, 0.3, and 0.4, the *F*1-score of the CNN model is higher than 94%. The ROC curve can show the influence of different thresholds on the generalization performance of the model, which is helpful to select the best threshold [22, 23]. We analyzed the ROC curve, compared the *F*1-score, and discussed with laparoscopy experts. Finally, we thought that when the confidence level was 0.4, the comprehensive performance of the model was more suitable for the dataset.

### 4.2. Medical Image Labeling Method

Using the correct labeling method is also an important aspect of the CNN model's target detection to achieve good results. Due to the complex environment of the endoscopic surgery, target detection in the endoscopic surgery is also a new challenge. There is currently no clear method for labeling the target tissue in the endoscopic surgery.

The article "Identification of the Vas Deferens in Laparoscopic Inguinal Hernia Repair Surgery Using the Convolutional Neural Network" was published in 2021. Journal: J Healthc Eng.

At the beginning of this study, when we labeled the vas deferens on the surgical images, because the features of the target do not take on a regular shape, in order to lessen the proportion of nonvas deferens tissue in the label box and reduce the influence of nonvas deferens tissue on the target tissue, we only labeled the area with obvious vas deferens features on the image. However, the results show that the model is unable to obtain all information pertaining to the vas deferens in these images, which leads to unsatisfactory training and testing results.

We adjusted the labeling method and expanded the scope of the label box so that the vas deferens tissue in the image could be included in the label box as much as possible. Although the proportion of the nonvas deferens in the label box increases, when we use the same training image and validation image and the same training parameters to train and test the model again, the training process and results show that the training effect of the new labeling method is better than our previous labeling method. The example after adjusting the labeling method is shown in line 2 of Figure 3, and the data details of the training process are shown in Figure 6.

Through the observation of the model training process, it is not difficult to find that different annotation methods will significantly affect the training effect of the model. During surgery, although the target tissue may be partially occluded by other nontarget tissues, our suggestion is to label the target tissue as completely as possible.

### 4.3. Indicator IoU and AP

IoU is the ratio of the overlap area and the union area of the label box and the test box. In the field of medical image recognition, the higher the IoU is, the higher the positioning accuracy is and the more it meets the needs of clinicians.

We tested the performance of the model under different IoU thresholds (0.7 to 0.2). The results showed that AP increased from 36.97% to 95.64%, and PPV increased from 58.82% to 99.82%.

We discussed with laparoscopic experts whether these labeled areas are enough to remind surgeons to identify the vas deferens. Experts believe that, in laparoscopic surgery, the role of computer-aided surgery is to remind surgeons to readily discover target tissue and to pay more attention to this target area. When surgeons know the general location of the vas deferens, they will be more alert and cautious, so as not to damage the vas deferens and other target tissues during surgery.

By comparing the images in the test results, experts believed that when the IoU was greater than 0.3, the labeling result was acceptable. However, when the IoU dropped to 0.2, some labels were inaccurate, the proportion of target tissue in the label box was too low to correctly represent the vas deferens, and the center of the label box was not located over the vas deferens. These results also tell us that IoU is also an important indicator to evaluate the performance of the model, and higher IoU will better assist doctors to observe and discover target organizations.

The article "Identification of the Vas Deferens in Laparoscopic Inguinal Hernia Repair Surgery Using the Convolutional Neural Network" was published in 2021. Journal: J Healthc Eng.

We found that when the IoU threshold was greater than 0.2, the TPR was lower than 90%, which indicated that the label box given by the model was not accurate enough, and the learning of the vas deferens was not enough. Although the model could recognize obvious features of the vas deferens, if the vas deferens' surface was partially obscured, the model could not accurately recognize and label the vas deferens. The details are shown in Figure 7.

### 4.4. Limitations

We used the CNN model to identify the vas deferens in laparoscopic inguinal hernia repair for the first time. Although we achieved satisfactory results, our research also has some limitations. First, we should further expand the number of patients and the absolute number of vas deferens images as the training dataset so that the CNN model can fully learn the characteristics of the vas deferens. Second, more indicators and test data should be set to evaluate the performance of the model, and we need to compare the performance with surgeons in different levels, so as to make the evaluation of the model more objective. Third, we only use the data of one hospital to train and verify the model, and the multicenter data will more effectively prove the detection and generalization ability of the model. Fourth, this model has a large number of parameters. Although the detection performance is satisfactory, it requires high computer configuration and time-consuming training process. We should further optimize the model structure, reduce the model parameters, and improve the model detection ability.

In future studies, we plan to collect more data from more hospitals, compare the neural network with the indicators of identifying important tissues in laparoscopic inguinal hernia repair by surgeons with different levels of experience, and further test whether this technology can help young general surgeons optimize the learning curve and reduce the incidence of vas deferens injury complications.

## 5. Conclusion

As an effective target detection method, computer deep learning technology has been widely used in medical image recognition [24–27]. In this study, we used YOLO (v4) to identify vas deferens images under laparoscopic inguinal hernia repair. We used different confidence levels from 0.1 to 0.9 to calculate various evaluation indicators in the image test dataset; picked the best confidence level for the video test dataset; adjusted the IoU thresholds from 0.2 to 0.7 to understand the positioning accuracy and AP of the model; and discussed with laparoscopic experts to select appropriate parameters to evaluate the performance of the model. In the image test dataset, the values of TPR, TNR, PPV, ACC, and *F*1 were 90.61%, 98.67%, 98.57%, 94.61%, and 94.42% (confidence level 0.4), respectively. In the video test dataset, the values of TPR, TNR, PPV, and ACC were 90.11%, 95.76%, 95.52%, and 92.93%, respectively. In IoU 0.3, the average precision (AP) was 92.38%.

The article "Identification of the Vas Deferens in Laparoscopic Inguinal Hernia Repair Surgery Using the Convolutional Neural Network" was published in 2021. Journal: J Healthc Eng.

We confirmed that a CNN can identify and label vas deferens images efficiently in laparoscopic inguinal hernia repair. This will help laparoscopic surgeons, especially young ones, to better carry out clinical work, optimize the learning curve of the laparoscopic surgery, improve surgical efficiency, and reduce surgical complications.

## Figures and Tables

**Figure 1:** Patient age distribution.

**Figure 2:** Research flowchart.

**Figure 3:** Original images. The first row shows original images with the vas deferens; the second row shows labels included by the experts; the third row shows original images without the vas deferens.

**Figure 4:** CNN-labeled vas deferens area and corresponding confidence level. The first row shows the true positive (TP); the vas deferens is labeled with a purple rectangle, and the confidence level is shown above the rectangle. The second line shows the false positive (FP). The third line shows the false negative (FN). The model does not give any labels on the image. The researchers circled the area of the vas deferens in yellow.

**Figure 5:** The ROC curve and AUC value.

**Figure 6:** Processes of training and validation using different labeling methods. (a) The graph showing the training process of the partial labeling method. (b) The graph showing the training process of the new labeling method. The red line shows the internal validation precision, and the blue line shows the loss curve.

**Figure 7:** The AP of the model under different IoU values and the corresponding image examples. In the first row and the third row, from left to right, AP curves at IoU 0.2 to 0.4 and 0.5 to 0.7 are shown. In the second row and the fourth row, the corresponding images at different IoU values are shown. The blue rectangle boxes were labeled by laparoscopic experts in advance, and the green rectangle boxes were labeled by the model.

The article "Identification of the Vas Deferens in Laparoscopic Inguinal Hernia Repair Surgery Using the Convolutional Neural Network" was published in 2021. Journal: J Healthc Eng.

**Table 1:** Dataset and patient information.

Dataset	Number of patients	Age (years)	Number of images
Training	26	63.15 ± 7.64	2,600
Image test	6	64 ± 8.12	1,200
Video test	3	55 ± 6.56	5,433

All patients are male.

**Table 2:** The test result at different confidence levels.

Confidence level	TP	FP	TN	FN
≥0.1	577	56	544	30
≥0.2	565	32	568	42
≥0.3	555	17	583	52
≥0.4	550	8	592	57
≥0.5	545	4	596	62
≥0.6	531	2	598	76
≥0.7	516	1	599	91
≥0.8	494	0	600	113
≥0.9	461	0	600	146

These results are based on all the detection boxes.

**Table 3:** The evaluation indicators at different confidence levels.

Confidence level	TPR (%)	TNR (%)	PPV (%)	ACC (%)	*F*1 (%)
≥0.1	95.06	90.67	91.15	92.87	93.06
≥0.2	93.08	94.67	94.48	93.87	93.85
≥0.3	91.43	97.17	97.03	94.28	94.16
≥0.4	90.61	98.67	98.57	94.61	94.42
≥0.5	89.79	99.27	99.27	94.53	94.29
≥0.6	85.01	99.62	99.62	93.54	93.16
≥0.7	85.01	99.81	99.81	92.38	91.82
≥0.8	81.38	100	100	90.64	89.73
≥0.9	75.95	100	100	87.9	86.33

**Table 4:** The evaluation indicators under different IoUs.

IoU	TPR (%)	PPV (%)	AP (%)	*F*1 (%)
≥0.2	88.73	99.82	95.64	93.95
≥0.3	87.75	98.71	92.38	92.91
≥0.4	85.95	96.69	89.31	91.00
≥0.5	80.72	90.81	80.88	85.47
≥0.6	72.22	81.25	68.73	76.47
≥0.7	52.29	58.82	36.97	55.36

These evaluation indicators are calculated based on 600 positive data items in the test dataset.

**Table 5:** The test results in the video test dataset.

Patients	TPR (%)	TNR (%)	PPV (%)	ACC (%)
1	90.23 (822/911)	96.14 (872/907)	95.92	93.18
2	89.50 (810/905)	95.23 (859/902)	94.96	92.36
3	90.58 (818/903)	95.91 (868/905)	95.67	93.25
Average	90.11 (2450/2719)	95.76 (2599/2714)	95.52	92.93

These evaluation indicators are calculated based on confidence level 0.4.

## Data Availability

The image and video data used to support the findings of this study are restricted by the Ethics Committee at Hannan Hospital in order to protect patient privacy.
